This article has been retracted.

# The Molecular Mechanism of Hepatic Lipid Metabolism Disorder Caused by NaAsO_2_ through Regulating the ERK/PPAR Signaling Pathway

**DOI:** 10.1155/2022/6405911

**Published:** 2022-03-14

**Authors:** Liping Wu, Shuling Zhang, Qi Zhang, Shaofeng Wei, Guoze Wang, Peng Luo

**Affiliations:** ^1^The Affiliated Hospital of Guizhou Medical University & Key Laboratory of Environmental Pollution Monitoring and Disease Control, Ministry of Education, School of Public Health, Guizhou Medical University, Guiyang 550025, China; ^2^State Key Laboratory of Functions and Applications of Medicinal Plants, Guizhou Medical University, Guiyang 550014, China; ^3^Guizhou Provincial Engineering Research Center of Food Nutrition and Health, Guizhou Medical University, Guiyang 550025, China

## Abstract

Chronic arsenic exposure is a risk factor for human fatty liver disease, and the ERK signaling pathway plays an important role in the regulation of liver lipid metabolism. However, whether ERK plays a role in the progression of arsenic-induced liver lipid metabolism disorder and the specific mechanism remain unclear. Here, by constructing a rat model of liver lipid metabolism disorder induced by chronic arsenic exposure, we demonstrated that ERK might regulate arsenic-induced liver lipid metabolism disorders through the PPAR signaling pathway. Arsenic could upregulate the expression of PPAR*γ* and CD36 in the rat liver, decrease the expression of PPAR*α* and CPT-1 in the rat liver, increase the organ coefficient of the rat liver, decrease the content of TG in rat serum, and promote fat deposition in the rat liver. In the arsenic-induced rat model of hepatic lipid metabolism disorder, we found that the expression of *p*-ERK was increased. In order to further explore whether the ERK signaling pathway was involved in arsenic-induced liver lipid metabolism disorder, we exposed L-02 cells to different arsenic concentrations, and the results showed that arsenic significantly increased the expression of P-ERK in L-02 cells in a dose-dependent manner. We further treated L-02 cells with ERK inhibitors and found that the expression of TG, PPAR*α*, and CPT-1 in L-02 cells increased, while the expression of P-ERK, PPAR*γ*, and CD36 decreased. In conclusion, ERK may be involved in arsenic-induced liver lipid metabolism disorder by regulating the PPAR signaling pathway. These findings are expected to provide a new targeting strategy for arsenic-induced liver lipid metabolism disorder.

## 1. Introduction

Arsenic is a common environmental poison, which is ubiquitous in water, coal, air, soil, and food. Its derived compounds can cause damage to the human skin, liver, lung, kidney, and other organs and cause diabetes, neurological diseases and various forms of cancer, cardiovascular and peripheral vascular diseases, and other diseases [1–5]. Although the incidence of arsenic exposure disease can be slightly reduced through health education, prohibition of the collection of high-arsenic coal, and renovation of stove facilities, the pathogenic mechanism of arsenic is unclear. Therefore, it is very important to study the pathogenic mechanism of arsenic and identify possible regulatory targets.

The liver is one of the main target organs of arsenic poisoning [6]. Previous studies have shown that chronic arsenic exposure can cause liver injury, hepatitis, liver fibrosis, cirrhosis, liver cancer, and other related malignant diseases [7, 8]. Population epidemiological investigations and experimental studies have confirmed that arsenic can cause liver damage. The liver damage caused by arsenic is mainly involved in lipid peroxidation, oxidative damage, DNA damage, inflammatory reaction, immune dysfunction, cell necrosis, and apoptosis [9–11]. The liver is the central metabolic organ of the human body and plays a momentous role in lipid metabolism; long-term accumulation of arsenic in the liver will lead to cell dysfunction and lipid metabolism disorder in the liver and result in the excessive lipid deposition in the hepatocytes [12]. Lipid deposition was mainly due to the increase in free fatty acid (FFA) transport to the liver, the high lipid diet, and the mobilization of peripheral adipose tissue; the *β*-oxidation of FFA was decreased in mitochondria of hepatocytes, resulting in the increase in TG; the synthesis of FFA and TG was increased in the endoplasmic reticulum of hepatocytes; deficient synthesis or secretion of very low-density lipoprotein (VLDL) resulted in reduced TG transport from inside to outside of liver cells [13]. The imbalance of synthesis, degradation, and secretion of liver lipid metabolism further led to abnormal deposition of lipid in liver cells [14]. Our previous study found that arsenic could cause lipid metabolism disorder in the process of hepatocyte injury [15]. Related research [16] had shown that there was a positive correlation between urinary arsenic exposure and nonalcoholic fatty liver disease (NAFLD) risk in American adolescents and adults, and arsenic exposure might be a risk factor for human fatty liver. Chronic arsenic exposure could aggravate the liver damage induced by high-fat diet in mice [17, 18]. However, the specific mechanism of arsenic-induced hepatic lipid metabolism disorder was not clear.

Sterol regulatory element-binding protein (SREBP) is a transcription factor family about cholesterol, and it has a significant role in the process of lipid metabolism and fatty acid and triglyceride biosynthesis controlling the expression of lipid synthesis and upstream gene [19, 20]. SREBP is composed of SREBP-1a, SREBP-1c, and SREBP-2. Among them, SREBP-1c mainly regulates the gene expression which regulates FA synthesis and is distributed in the liver [21]. By regulating the expression of fatty acid synthase (FASN), it could increase lipid synthesis in the liver [22].

Peroxisome proliferator-activated receptor (PPAR) is a member of the nuclear receptor transcription factor superfamily consisting of PPAR*α*, PPAR*β*/*δ*, and PPAR*γ*. Among them, PPAR*α* is the main regulatory protein involved in liver *β*-oxidation, which can control the *β*-oxidation of fatty acid (FA) in mitochondria by regulating the downstream target gene carnitinepalmitoyltransferase1 (CPT1) [23]. In hepatocytes, PPAR*γ* was a regulator of lipid metabolism, targeted to participate in FA introduction, promoted fatty acid transporter- (FAT/CD36) mediated FFA uptake, and promoted the increase in triglycerides in the liver [24]. In the research of a nonalcoholic fatty liver model established by high-fat diet, it was found that the expression of PPAR*α* and its downstream genes both decreased. The *β*-oxidation level of FA in hepatocytes decreased; as a result, the FA accumulated in cells, while the expression of PPAR*γ* and its downstream genes increased, which increased the content of FFA in cells and aggravate nonalcoholic fatty liver further [25]. Existing studies had found that the mitogen-activated protein kinase (MAPK) signaling pathway was related to lipid metabolism [26]; the molecular mechanism of the MAPK signaling pathway regulating fat metabolism might be related to PPAR*α*, SREBP-1, and diacylglycerol acyltransferase (DGAT).

Extracellular signal-regulated kinase (ERK) is one of the pathways of MAPK, which plays an important role in proliferation, differentiation, and apoptosis [27]. Existing studies had found that the ERK signaling pathway was related to lipid metabolism. Preadipocytes regulated its differentiation positively and negatively by regulating lipid metabolism-related genes such as PPARs and SREBP-1c [28, 29]. In algae cells, the accumulation of intracellular lipids was promoted by activating ERK, and the intracellular lipid content decreased after the treatment with the ERK-specific inhibitor PD98059 [29]. In the previous study of our group, we found that arsenic could cause liver injury and liver fibrosis through the ERK signaling pathway. In summary, by combining previous studies on the ERK signaling pathway and arsenic-induced liver injury, we were interested in whether the ERK signaling pathway plays a role in arsenic-induced liver lipid metabolism disorder and its specific mechanism.

Therefore, in order to clarify the mechanism of arsenic-induced liver lipid metabolism disorder and explore the role of ERK regulating the PPAR signaling pathway in arsenic-induced liver lipid metabolism disorder, we explored the causes of arsenic-induced liver lipid metabolism disorder by using molecular biology- and toxicology-related experimental techniques *in vivo* and *in vitro*. These data would provide some new perspectives and targets for the treatment of arsenic-induced liver lipid metabolism disorder.

## 2. Materials and Methods

### 2.1. A Model of Arsenic-Induced Hepatic Lipid Metabolism Disorder in SD Rats

Male SD rats (80-100 g, without specific pathogens) were provided by the Experimental Animal Center of the Third Military Medical University. In order to investigate the effect of NaAsO_2_ (Sigma Chemical Corp, USA) on the rat liver, the SD rats were fed with 50 mg/kg arsenic diet by intragastric administration for 5 months; the control group was fed with basic feed as a carrier.

### 2.2. The Construction of Arsenic-Induced In Vitro Cell Model

L-02 cells were provided by the Cell Bank of Chinese Academy of Sciences (Shanghai). 1% penicillin/streptomycin and 10% fetal bovine serum were added to the DMEM medium and cultured at 37°C in a wet incubator containing 5% CO_2_. To prepare the original solution (10 mM), 129.91 mg NaAsO_2_ was dissolved in 100 ml double distilled water. L-02 cells were exposed to 0 (control group), 8 *μ*M, 16 *μ*M, and 32 *μ*M NaAsO_2_ for 24 h; the concentration of NaAsO2 was obtained through the previous study of our research group [15]. L-02 cells were pretreated with 10 *μ*M ERK inhibitor (PD98059, MCE) for 4 h and then cultured with 16 *μ*M NaAsO_2_ for 24 h.

### 2.3. Organ Coefficient Detection and Histopathological Examination

At the end of the fifth month, the SD rats were euthanized. The corresponding value was obtained by comparing with the body weight of rats. In liver histological analysis, the SD rats' liver tissue was fixed in 4% paraformaldehyde, embedded in paraffin, and stained with hematoxylin and eosin (HE), and the expression of related proteins was observed by immunohistochemistry (IHC). The results were obtained by microscope analysis.

### 2.4. The Detection of TG and Oil Red O Staining of SD Rat Serum, Liver Tissue, and L-02 Cells

The blood was taken from the heart, and the supernatant was obtained by centrifugation at 4°C for 5 min, at the rate of 3500 rpm/min. The absorbance was measured by the glycerol-3-phosphate oxidase method and with a spectrophotometer at 546 nm wavelength. The SD rats' liver tissue sections were fixed with formaldehyde for 10 min and washed with distilled water for 3 times and 60% isopropanol. After the liver tissue sections were dehydrated, they were smeared with oil red O for 10 minutes and rinsed with distilled water for 3 times. Glycerol-sealed tablets were observed under a microscope. L-02 cells were treated with cell lysate, according to the instructions of the Nanjing built triglyceride assay kit; L-02 cells were added to a 96-well plate with 3 wells in each group, and the OD value (550 nm) was determined by using an enzyme labeling instrument. L-02 cells were counted as 1 × 10^5^ cells per well, and 24-well plates were taken for plate laying. Discard the medium, add PBS to gently wash off the residual medium, and 4% paraformaldehyde was used for fixation for 30 min. Rinse with PBS for 2-3 times, dye with oil red O staining solution for 30 min, and then wash with PBS for 1-2 times. The staining was observed by using a white light microscope, and the red staining was a lipid-positive staining area.

### 2.5. Quantitative Real-Time PCR (qRT-PCR) of Protein Coding Genes Related to Lipid Metabolism

Use the TRIzol Reagent (Tiangen Technology Co., Ltd.) to extract total RNA from SD rats' liver tissue and L-02 cells, according to the instructions of the Takara reverse transcription kit, and the sample system was used to expand the proportion according to the need to synthesize cDNA. SREBP-1c, FASN, PPAR*α*, CPT-1, PPAR*γ*, CD36, and internal reference genes (GAPDH, *β*-actin) were analyzed according to the scheme provided by the manufacturer. qRT-PCR analysis was performed using the CFX-96 real-time fluorescence quantitative PCR instrument (Bio-Rad Company, USA) and SYBR Premix Ex Taq HS qPCR kit (Takara Company). The relative expression of the target gene was obtained by delta 2^−△△ct^ method. Primers are provided in Tables 1 and 2.

### 2.6. Western Blotting Assay of Proteins Related to Lipid Metabolism

RIPA lysate F (Beyotime, Shanghai, China) was used to extract protein from SD rats' liver tissue and L-02 cells. The total protein concentration was determined by using the BCA kit (Solebo Company). SREBP-1c, FASN, PPAR*α*, CPT-1, PPAR*γ*, and CD36 were analyzed. The same amount of protein in liver tissue and L-02 cells was separated by using the SDS-PAGE kit (Shanghai Biyuntian Company) and transferred to the polyvinylidene fluoride (PVDF) membrane (Bio-Rad Company). The cell membrane was sealed with 5% skim milk for 2 h, incubated overnight with different antibodies, and incubated with horseradish peroxidase-labeled disomic for 1 h, and the protein expression level was detected by using the ECL kit (Millipore Company, USA). The antibody reactivity was detected by using the ECL Western blotting detection system. The density of protein bands was analyzed by using ImageJ software (Bio-Rad, California, USA).

### 2.7. Statistical Analysis

SPSS 20.0 statistical software was used for statistical analysis. The data were tested by the normality test and variance homogeneity test, and the results were expressed as mean ± standard deviation (SD). Single-factor analysis of variance (ANOVA) was used to compare the mean among groups. The LSD method was used for further pairwise comparison, and the Games-Howell method was used for variance discrepancy. *P* < 0.05 indicates that the difference was statistically significant.

## 3. Results

### 3.1. Establishment of a Rat Model of Arsenic-Induced Lipid Disorder

In order to determine the relationship between arsenic and liver lipid metabolism, we first constructed *in vivo* samples of SD rats and observed the effects of NaAsO_2_ on the SD rat liver by detecting organ coefficient, TG content, HE staining, and oil red O staining. The results showed that the liver organ coefficient of SD rats fed with NaAsO_2_ and the degree of steatosis and lipid aggregation in liver tissue were significantly increased (Figure 1(a)), the serum TG content was decreased (Figure 1(b)), lipids in liver tissue showed orange color (Figure 1(d)), and optical density was increased (Figure 1(e)). These results indicated that the model of liver lipid metabolism disorder induced by arsenic had been established successfully.

### 3.2. NaAsO_2_ Exposure Increased the Level of Lipid Transport and Decreased the Level of Lipid Oxidation and Lipid Synthesis in the SD Rat Liver

To further verify the effects of arsenic on lipid metabolism in the rat liver, we detected the expressions of PPAR*γ*, CD36, PPAR*α*, CPT-1, SREBP-1C, and FASN in the NaAsO_2_ group. qRT-PCR results showed that NaAsO_2_ could increase the expression of PPAR*γ* and CD36 mRNA in the SD rat liver and decrease the expression of PPAR*α*, CPT-1, SREBP-1c, and FASN (Figure 1(h)). IHC and Western blotting results showed that the expression levels of PPAR*γ* and CD36 were increased and the expression levels of PPAR*α*, CPT-1, SREBP-1c, and FASN were decreased (Figures 1(f), 1(i), and 1(j)). These results suggested that NaAsO_2_ exposure could increase the level of lipid transport and decrease the level of lipid oxidation in the SD rat liver.

### 3.3. Increase in p-ERK Protein in the Rat Liver Induced by NaAsO_2_ Exposure

Based on our previous findings, the ERK signaling pathway was involved in arsenic-induced apoptosis and mitochondrial autophagy. In order to have a deep understanding of the mechanism of the ERK signaling pathway and arsenic, we further explored the expression of ERK in arsenic-induced liver lipid metabolism disorders. Western blotting was used to detect the expression of *p*-ERK and ERK proteins in the rat liver. The results showed that the expression level of *p*-ERK protein and the ratio of *p*-ERK/ERK protein content in the NaAsO_2_ group were significantly higher. To sum up, NaAsO_2_ exposure induced the activation of the ERK signaling pathway in the rat liver (Figure 1(i)).

The *in vivo* experiments showed that NaAsO_2_ could lead to hepatic lipid metabolism disorder and then trigger fat accumulation causing fatty liver, mainly by promoting FFA to intracellular transport, inhibiting fatty acid oxidation, and TG transport to the periphery. However, NaAsO_2_ could inhibit the synthesis of intracellular TG by inhibiting the expression of SREBP-1c and its downstream genes. At the same time, NaAsO_2_ could increase the expression of *p*-ERK protein in the SD rat liver, in order to further clarify the effect of arsenic exposure on hepatocytes and explore the role of ERK in hepatic lipid metabolism. In the next step, we would select L-02 cells at the cellular level for in-depth study.

### 3.4. The Role of ERK in Lipid Metabolism Disorder Induced by NaAsO_2_ Exposure in L-02 Cells

To further confirm the potential mechanism of the ERK signaling pathway in arsenic-induced hepatic lipid metabolism disorder in SD rats, we constructed an *in vitro* experiment with L-02 cells as the research object and observed the expression of *p*-ERK by poisoning L-02 cells with different arsenic concentrations. The results showed that *p*-ERK expression was increased with the increase in NaAsO_2_ concentration. With the aim of further exploring the role of the ERK signaling pathway in the arsenic-induced lipid metabolism of L-02 cells, we treated L-02 cells with a powerful inhibitor PD98059 (10 *μ*M) for 4 h and then with arsenic (16 *μΜ*) for 24 h. Western blotting results showed that *p*-ERK protein expression in the ERK inhibitor group was significantly lower than that in the NaAsO_2_ group (Figures 2(a) and 2(b)).

### 3.5. ERK Inhibited the Content of TG in L-02 Cells Exposed to NaAsO_2_

To understand whether the ERK signaling pathway regulates arsenic-induced liver lipid metabolism disorders, we intervened with L-02 cells by using the ERK effective inhibitor PD98059. By TG content detection and oil red O staining observation in L-02 cells, compared with the control group, the TG content was decreased, and the orange fat particles were decreased in the NaAsO2 group. After PD98059 intervention, compared with the NaAsO_2_ group, TG content and fat particles were increased in L-02 cells. In conclusion, the ERK signaling pathway inhibited the TG content in L-02 cells under the action of NaAsO_2_ (Figures 2(c) and 2(d)).

### 3.6. ERK Targeting the PPAR Signaling Pathway Promoted the Expression of Lipid Transport Genes and Restrained the Lipid Oxidation Gene Expression in L-02 Cells Exposed to NaAsO_2_

In order to further elucidate that arsenic-induced hepatic lipid metabolism disorder was regulated by ERK, we observed the changes of hepatic plasma metabolism genes in arsenic-poisoned L-02 cells after PD98059 intervention by qRT-PCR and Western blotting. The results showed that the expressions of PPAR*γ* and CD36 mRNA and PPAR*γ* protein were increased in L-02 cells in the NaAsO_2_ group and the expressions of PPAR*α*, CPT-1, SREBP-1C, and FASN mRNA and PPAR*α* and SREBP-1c proteins were decreased, compared with the control group. After treatment with PD98059, compared with the NaAsO_2_ group, the expression levels of PPAR*γ* and CD36 mRNA and PPAR*γ* protein were decreased and the expression levels of PPAR*α* and CPT-1 mRNA and PPAR*α* protein were increased. Interestingly, the expression of SREBP-1c and FASN mRNA and SREBP-1c protein decreased, and the difference was not statistically significant. These results suggested that the ERK signaling pathway mediated NaASO_2_-induced liver lipid metabolism disorders by regulating PPAR-related genes (Figures 2(e), 2(f), and 2(g)).

## 4. Discussion

Arsenic is an environmental poison and known as a human carcinogen that seriously harms human health. Its derivative compounds cause not only skin lesions [16] and peripheral nervous system injury [17] but also liver injury, liver fibrosis, cirrhosis, and liver cancer [25, 30]. In the study of population exposed to high arsenic concentration in the environment of exposed workers, the detection rate of fatty liver and liver enlargement was obviously higher than that of control group unexposed to arsenic environment [31, 32]; it showed that arsenic exposure might be a risk factor for human fatty liver disease, but the specific mechanism of arsenic to liver lipid metabolism disorder was unclear. In this study, we explored the mechanism of arsenic-induced hepatic lipid metabolism disorder *in vivo* and *in vitro*.

The liver is one of the main metabolic organs of the human body and also one of the target organs of arsenic [6]. Long-term accumulation of arsenic in the liver will cause not only liver injury, liver fibrosis, liver apoptosis, etc., but also liver lipid metabolism disorder, resulting in excessive deposition of lipid in the liver [17, 32]. In this study, the SD rats were fed with NaAsO_2_, and the results showed that the organ coefficient and the fat particles of the liver were increased in the NaAsO_2_ exposure group, which indicated that NaAsO_2_ would cause hypertrophy and lipid accumulation in the liver. Other studies have found that arsenic exposure will aggravate liver damage in mice fed with high-fat diet and arsenic [17, 18], which is consistent with the results of this study and further confirms that arsenic may lead to the occurrence of fatty liver. However, the results of the SD rats fed with NaAsO_2_ showed that the decrease in TG content might indicate arsenic damage to SD rats' liver, resulting in insufficient synthesis or secretion of very low-density lipoprotein (VLDL), and reduced TG transport from inside to outside the liver cells, which might cause imbalance in synthesis, degradation, and secretion of liver lipid metabolism, causing abnormal deposition of lipids in liver cells. Arsenic trioxide had a significant effect on the treatment of acute promyelocytic leukemia [33]; interestingly, triglyceride levels were increased during treatment [34], so the specific mechanisms of arsenic and triglyceride needed to be further studied.

Meanwhile, NaAsO_2_ exposure significantly reduced TG content and fat particles in L-02 cells. Paradoxically, the results *in vivo* and *in vitro* were inconsistent. The reason might be that the study in this cell experiment only covered the effects of arsenic on the lipid metabolism of cells, including the de novo lipid synthesis level, lipid oxidation, and lipid output, which could not completely simulate normal physiological functions of the body and failed to involve the effects of NaAsO_2_ on the absorption and circulating lipid level of the liver. Existing studies had shown that arsenic could cause an increase in serum FFA content [35], and circulating lipids could not be absorbed in vitro experiments, which might be the reason for the inconsistent results between *in vitro* and *in vivo* experiments. The results of this study suggested that in a separate experiment *in vitro*, NaAsO_2_ could reduce intracellular TG content in one or more ways from de novo lipid synthesis, lipid oxidation, and lipid output levels.

SREBP is a kind of membrane connexin located in the endoplasmic reticulum, which is an important regulator of lipid synthesis in animals [19, 20]. It promoted the synthesis of cholesterol, fatty acids, and triglycerides, by regulating the gene transcription of enzymes related to lipid production. In an *in vivo* experiment of this study, it was found that the expression levels of SREBP-1c and its downstream target gene FASN were lower in the NaAsO_2_ group than in the control group. In addition, the content of TG in cells decreased with the increase in arsenic exposure dose. In the study of lipid metabolism in mice exposed to low-dose arsenic, it was found that chronic arsenic exposure could induce the decrease in SREBP-1c expression in the liver, which decreased TG synthesis in hepatocytes [36], and it was consistent with the results of this study. Although the expression levels of SREBP-1c and its downstream gene FASN were decreased, hepatocyte steatosis still occurred in animal experiments. It was suggested that NaAsO_2_ inhibited the expression of SREBP-1c, which related to ab initio lipid synthesis and the expression of FASN and its downstream gene. NaAsO_2_ may cause hepatic steatosis in the *in vivo* experiment, which provided a new target for arsenic as a treatment of triglyceride oversynthesis caused by high-fat diet.

PPAR*α* is the main regulator of liver *β-*oxidation and microsomal *ω* oxidation, and CPT-1 is its downstream gene [37]. In the study of nonalcoholic fatty liver, it has been found that inhibiting the expression of PPAR*α* and its downstream genes in the liver could reduce the *β*-oxidation of fatty acids and promote the accumulation of fatty acids in the liver [38, 39]. The *in vivo* experiment of this study found that the expression of the PPAR*α* gene was lower in the NaAsO_2_ group than in the control group, which indicated that NaAsO_2_ inhibited the *β-*oxidation of fatty acids in hepatocytes and promoted the accumulation of lipids in the liver [40, 41]. In the *in vitro* experiment, the expression of the PPAR*α* gene in the NaAsO_2_ group was also lower than that in the control group, indicating that its expression was dose-dependent. Therefore, NaAsO_2_ inhibited the *β*-oxidation of fatty acids in hepatocytes, and the expression level of PPAR*α* was also related to the level of lipid output, which positively regulated MTTP. The results showed [42] that the expression of MTTP was decreased, when the expression of PPAR*α* was decreased. However, MTTP is the key component of intracellular TG output, which leads to a decrease in the output of TG to the periphery, and it is also consistent with the results of serum TG detection in the *in vivo* experiment. In this study of the *in vitro* experiment, we found that NaAsO_2_ inhibited the expression of the fat synthesis gene SREBP-1c and decreased triglyceride synthesis in hepatocytes. Although NaAsO_2_ also inhibited the expression of the fatty acid oxidation gene PPAR*α*, it could not induce fat accumulation in hepatocytes. It was suggested that although NaAsO_2_ inhibited the *β*-oxidation of fatty acids and the peripheral transport of TG, it might not be the main factor of fatty liver degeneration caused by NaAsO_2_.

PPAR*γ* is the main gene regulating lipid synthesis, which affects the transport of extracellular free fatty acids to cells by regulating the expression of its downstream gene CD36 [43]. In the *in vivo* experiment of this study, it was found that the expression levels of PPAR*γ* and CD36 proteins and mRNA were higher in the NaAsO_2_ group than in the control group, and the results were consistent with those in the *in vitro* experiment, indicating a dose-dependent manner. Therefore, NaAsO_2_ promoted the transport of free fatty acids to cells by activating the PPAR*γ* pathway, which led to hepatocyte steatosis. It had been found that arsenic enhances lipolysis of adipocytes through the GPCR pathway and increased the content of FA in circulation [44]. Combined with the research, it could be shown that NaAsO_2_ increased the content of FFA in the blood by promoting the oxidation of adipose tissue and promoted its transport and accumulation to other nonadipose tissue, which led to fat deposition. It was known that NaAsO_2_ promoted lipolysis of adipose tissue, increased the release of FA, and promoted the transport of free fatty acids to cells by activating the PPAR*γ* pathway, resulting in hepatocyte steatosis. To sum up, NaAsO_2_ exposure could induce the disturbance of hepatic lipid metabolism, probably by promoting FA uptake and inhibiting TG transport to the periphery.

The ERK signaling pathway is one of the pathways of MAPK, which mainly regulates cell proliferation, differentiation, and apoptosis [45–47]. Related studies had shown that [48, 49] the MAPK pathway participated in glucose and lipid metabolism in the liver. In preadipocytes, the *P*38 signaling pathway improved the antioxidant capacity of the liver, regulated apoptosis and autophagy of liver cells, and alleviated liver inflammation and injury [50]. The ERK signaling pathway could induce the expression of lipid metabolism-related genes such as PPARs and SREBP-1c, which positively and negatively regulated preadipocyte differentiation [9, 28]. The accumulation of intracellular lipids was promoted by activating the ERK signaling pathway, and the intracellular lipid content was decreased after the treatment with the ERK-specific inhibitor PD98059 [29]. Although a large number of data had been proven in the study of hepatitis [51, 52], the role of ERK in lipid metabolism was not clear.

Based on our previous findings, the ERK signaling pathway was involved in arsenic-induced liver fibrosis [53] and L-02 cell apoptosis/autophagy [5]. In this study, in order to further explore the mechanism of the ERK signaling pathway in arsenic-induced liver injury, the ERK inhibitor was used to intervene with NaAsO_2_-exposed L-02 cells. The results of TG content detection and oil red O staining showed that the TG content of hepatocytes was increased in the ERK inhibitor group. Combined with the causes of hepatic steatosis caused by NaAsO_2_, the ERK signaling pathway might participate in lipid metabolism by regulating lipid synthesis, oxidative decomposition, and lipid transport. Other studies [54] had shown that ERK inhibits the expression of SREBP-1c in the model of nonalcoholic fatty liver induced by high-fat diet, and the MEK/ERK pathway played an important role in SREBP-1c expression induced by high-fat diet in NAFLD rats. In hepatoma cells, the ERK signaling pathway could reduce intracellular reactive oxygen species by inhibiting the expression of SREBP-1c [55], while in HACAT cells, the ERK inhibitor (PD98059) had no effect on the expression of SREBP-1c [56]. In our study, the expression of SREBP-1c was not significantly changed between the inhibitor group and the NaAsO_2_ group. Therefore, although NaAsO_2_ regulated the expression of ERK and SREBP-1c, the regulation of SREBP-1c by ERK was not significant.

NAFLD is a clinicopathological syndrome characterized by diffuse hepatocyte vesicular fat, which is caused by alcohol and other definite liver-damaging factors, including simple nonalcoholic fatty liver, nonalcoholic hepatitis, and liver cirrhosis to the final liver cancer [57]. The PPAR*α* pathway is involved in the regulation of fatty acid *β-*oxidation, inflammation, and liver cancer, while the ERK signaling pathway was also involved in the regulation of inflammation and liver cancer. Some studies had found that there was a correlation between ERK and PPAR*α* in hepatocytes; ERK participated in lipid metabolism by regulating PPAR*α* [58]. The results of this study showed that the inhibitor could decrease the expression of *p*-ERK protein and increase the expression of PPAR*α* and its downstream genes in L-02 cells exposed to NaAsO_2_. It is suggested that NaAsO_2_ can promote the phosphorylation of ERK and inhibit the oxidative decomposition of FA in cells by regulating the ERK pathway. In addition, it was found that in NAFLD, osteoprotegerin could regulate liver lipid metabolism by targeting the ERK/PPAR*γ*/CD36 pathway, and hypertension could be regulated by the ERK/PPAR*γ* signal pathway in cardiovascular disease [59]. In the results of this study, it was found that the expression levels of PPAR*γ*/CD36 were decreased after the action of the ERK inhibitor. This suggested that ERK affected hepatic lipid metabolism by regulating PPAR*γ*/CD36.

## 5. Conclusion

To sum up, combined with the experimental results *in vivo* and *in vitro*, we found that arsenic reduced the oxidation of FFA in hepatocytes by inhibiting the expression of PPAR*α* and its downstream genes. In addition, arsenic enhanced the uptake of FFA, inhibited the peripheral transport of TG, and resulted in lipid accumulation in the liver by promoting the expression of PPAR*γ* and CD36. Therefore, it was speculated that the mechanism of lipid metabolism accumulation induced by arsenic might be affected through activating the ERK/PPARs pathway, promoting FFA transport into cells, leading to lipid accumulation and lipid metabolism disorder in the liver. This finding further elucidates the molecular mechanism of arsenic-induced lipid metabolism disorder and provides an important molecular target for the prevention and treatment of arsenic-induced liver lipid metabolism disorder (Figure 3).

## Figures and Tables

**Figure 1:** Establishment of an SD rat model of arsenic-induced lipid disorder. NaAsO_2_ exposure could increase the level of lipid transport and decrease the level of lipid oxidation and lipid synthesis in the SD rat liver. *p*-ERK protein was increased in the SD rat liver by NaAsO_2_-induced exposure. (a) Liver coefficient of SD rats treated with NaAsO_2_. (b) TG of SD rats treated with NaAsO_2_. (c) HE staining in the liver of SD rats treated with NaAsO2. (d) Oil red O staining in the liver of SD rats treated with NaAsO_2_. (e) Oil red O staining value in the liver of SD rats treated with NaAsO_2_. (f) Immunohistochemical values in the liver of SD rats treated with NaAsO_2_. (g) mRNA expression in the liver of SD rats treated with NaAsO_2_. (h) Protein expression in the liver of SD rats treated with NaAsO_2_. (i) Protein bands in the liver of SD rats were treated with NaAsO_2_. (j) Liver immunohistochemistry of SD rats treated with NaAsO_2_.

**Figure 2:** The role of ERK in lipid metabolism disorder induced by NaAsO_2_ exposure in L-02 cells. ERK inhibited the content of TG which promoted the expression of lipid transport genes and restrained the inhibition of lipid oxidation gene expression in L-02 cells exposed to NaAsO2. (a) *p*-ERK protein expression of NaAsO_2_-infected L-02 cells. (b) *p*-ERK protein band of NaAsO_2_-infected L-02 cells. (c) PD98059 interfered with TG content of NaAsO_2_-infected L-02 cells. (d) PD98059 interfered with oil red staining of NaAsO_2_-infected L-02 cells. (e) PD98059 interferes with the expression of related mRNA in NaAsO_2_-infected L-02 cells. (f) PD98059 interfered with the expression of related protein in NaAsO_2_-infected L-02 cells. (g) PD98059 interfered with the expression bands of related protein in NaAsO_2_-infected L-02 cells.

**Figure 3:** The molecular mechanism of hepatic lipid metabolism disorder caused by NaAsO_2_ through regulating the ERK/PPAR signaling pathway.

**Table 1:** The primers of target genes in the animals for qRT-PCR.

Target gene		(5′-3′)
*β*-Actin	Forward	CCTAGACTTCGAGCAAGAGA
	Reverse	GGAAGGAAGGCTGGAAGA
FASN	Forward	GCAAAGCTGGTGTCATCC
	Reverse	CCTTAGTAGTGCGTGGTCG
CPT-1	Forward	GAGTCAAATGGGAAGGAAT
	Reverse	CAAGGCTACAATGGGACA
PPAR*γ*	Forward	CAATCTGCCTGAGGTCTG
	Reverse	TGGAGCCTAAGTTTGAGTT
PPAR*α*	Forward	TTCCTGCGAGTATGACCC
	Reverse	AAAACTGAAGGCAGAAATCC
CD36	Forward	TGTCTGGGTTCTGGAGTG
	Reverse	ATTGGGAAAGTTATTGCG
SREBP-1c	Forward	CCGAAGCATCAGAGGGAGT
	Reverse	GGATAACCAGGTGAAAGCC

**Table 2:** The primers of target genes in the L-02 cells for qRT-PCR.

Target gene		(5′-3′)
*β*-Actin	Forward	CTACCTCATGAAGATCCTCACCGA
	Reverse	TTCTCCTTAATGTCACGCACGATT
Fasn	Forward	TCGTGTTGACTTCTCGCTCC
	Reverse	TGCAGACGTCCTGGAAGAAC
CPT1	Forward	CCAGACGAAGAACGTGGTCA
	Reverse	ATCTTGCCGTGCTCAGTGAA
PPAR*α*	Forward	ACTGGCATTTGTTTCTGTT
	Reverse	CCTCGGTGACTTATCCTG
PPAR*γ*	Forward	AAATGCTGGAGAAGTCAA
	Reverse	AAAGAAGCCAACACTAAAC
CD36	Forward	GTCGGATTCAAATACAGC
	Reverse	TGTCCTATTGGGAAAGTC
SREBP-1	Forward	CTCACCAGGGTCGGCAAA
	Reverse	ACTTCATCAAGGCAGACTCGC

## Data Availability

All data required to evaluate the conclusions in this paper are included in this paper.
